This article has been retracted.

# Efficacy and Safety of Rupatadine Fumarate Combined with Acupoint Application in Allergic Rhinitis Complicated with Diabetes

**DOI:** 10.1155/2022/6935758

**Published:** 2022-06-14

**Authors:** Yu Liu, Pengjun Jiang, Xuqing Chen, Wen Zhang, Jun Shi

**Affiliations:** ^1^Department of Otolaryngology, Nanjing Integrated Traditional Chinese and Western Medicine Hospital Affiliated with Nanjing University of Chinese Medicine, Nanjing 210014, China; ^2^Department of Hematology, Affiliated Hospital of Nanjing University of Chinese Medicine, Nanjing 210029, China; ^3^Department of Otolaryngology, Affiliated Hospital of Nanjing University of Chinese Medicine, Nanjing 210029, China

## Abstract

The prevalence of allergic rhinitis has exhibited an upward trend, and diabetes is a common endocrine metabolic disorder. Treatment of allergic rhinitis complicated with diabetes has been marginally explored. This study aimed to observe the effect of rupatadine fumarate combined with acupoint application in the treatment of allergic rhinitis complicated with diabetes and its effect on serum IgE levels. Totally 80 patients with allergic rhinitis complicated with diabetes admitted to our hospital from December 2019 to December 2020 were recruited and assigned to receive either rupatadine fumarate (control group) or rupatadine fumarate plus acupoint application (research group). The clinical observation indexes of the two groups of patients before and after treatment were analyzed, and the clinical efficacy of the two groups was evaluated. Rupatadine fumarate plus acupoint application was associated with a significantly higher efficacy (23 cases of markedly effective, 14 cases of effective, and 3 cases of ineffective) versus rupatadine fumarate alone (14 cases of markedly effective, 16 cases of effective, and 10 cases of ineffective) (*χ*^2^ = 4.501, *p* = 0.034). The immunoglobulin E (IgE) and nasal mucosal eosinophils (EOS) levels of the two groups of patients after treatment decreased significantly, and the research group had lower results (*p* < 0.05). Patients in the research group showed significantly lower syndrome scores than those in the control group (*p* < 0.05). Rupatadine fumarate plus acupoint application resulted in significantly lower physical sign scores and interleukin-4 (IL-4) levels and higher levels of interferon-gamma (INF-*γ*) versus rupatadine fumarate alone (*p* < 0.05). The two groups showed a similar incidence of adverse events (*p* > 0.05). Rupatadine fumarate plus acupoint application may offer a viable alternative for the treatment of allergic rhinitis as it alleviates the clinical symptoms, improves the treatment efficiency, and enhances the anti-allergic effect of the drug, with a high safety profile.

## 1. Introduction

In recent years, the prevalence of allergic rhinitis has exhibited an upward trend due to environmental factors such as air pollution. Statistics show that the global incidence of the disease is 10–20% [1–3]. Diabetes may lead to allergic rhinitis due to impaired immune function [4]. At present, clinical treatment for allergic rhinitis is mainly based on antihistamines or corticosteroids [5]. However, the efficacy remains controversial in clinical settings since antihistamines and corticosteroids are associated with recurrence and adverse drug reactions [6].

Recently, traditional Chinese medicine (TCM) treatment has demonstrated great advantages in clinical medicine [7, 8]. Acupoint application is a treatment method guided by the basic theory of TCM, applying Chinese herbal preparations to the acupoints [9, 10]. Acupoint application therapy is used to stimulate the meridians, harmonize qi and blood, improve blood circulation, enhance immune function, and regulate the dynamic balance of the human body through acupoint stimulation [11]. TCM classifies allergic rhinitis into the category of *bi-qiu*, and acupuncture and acupoint application are frequently used for early treatment [12]. This study intends to combine acupoint application therapy with rupatadine fumarate to enhance the curative effect of allergic rhinitis and enrich the clinical data for the treatment of allergic rhinitis.

## 2. Materials and Methods

### 2.1. Inclusion Criteria

Patients who met the western medicine diagnostic criteria in *Guidelines for the Diagnosis and Treatment of Allergic Rhinitis* [13], TCM diagnostic criteria in *Guidelines for the Diagnosis of Common Diseases in TCM Otorhinolaryngology* [14], and diagnostic criteria for diabetes, aged >18 years old, with no recent use of anti-allergic rhinitis drugs two weeks prior to enrollment, who voluntarily participated in the study, with good treatment compliance, and with no allergies to the drugs used in this study were included.

### 2.2. Exclusion Criteria

Patients with severe systemic diseases, with allergic sinusitis, acute rhinitis, autonomic rhinitis, and other diseases, with allergic asthma, with communication impairments, cognitive disorders, or physical disabilities, during pregnancy or lactation, and with use of peripheral H1 receptor antagonist within 1 week before enrollment were excluded.

### 2.3. Screening and Grouping

Between December 2019 and December 2020, 80 patients with allergic rhinitis admitted to our hospital were considered eligible and recruited as per the inclusion and exclusion criteria. According to the treatment plan of the patients, they were equally assigned to a control group or a research group. This study is a retrospective analysis, does not interfere with the patient's treatment plan, and is supervised by the ethics committee of Affiliated Hospital of Nanjing University of Chinese Medicine, No. A-NJ1138.

### 2.4. Method

Patients in the control group received 10 mg rupatadine fumarate tablets (Yangzijiang Pharmaceutical Group Nanjing Hailing Pharmaceutical Co., Ltd., approval no. H20130047) daily after meals in the evening. A similar treatment protocol of rupatadine fumarate was introduced to the patients in the research group.

Patients in the research group received additional acupoint application. (1) Drug preparation: Corydalis, white mustard seeds, asarum, and raw kansui were ground into powder and mixed well at a ratio of 1 : 1 : 0.5 : 0.5, followed by the addition of ginger juice to make a herbal paste, and borneol and a small amount of vaseline were added to prepare a 1 cm × 1 cm × 0.5 cm medicinal pie. (2) The acupoint application was performed on the following acupoints of *Xinshu* (bilateral), *Feishu* (bilateral), *Geshu* (bilateral), *Shenshu* (bilateral), *Pishu* (bilateral), *Guanyuan*, and *Dazhui* using the prepared medicinal cakes. (3) Application method: the medicinal cakes were applied to the corresponding acupoints, fixed with a 5 cm × 5 cm desensitizing tape and removed after 8 hours. The skin of the application site should be protected from water for 24 hours. The acupoint application was performed once per week, with four weeks as a course of treatment. (4) Precautions: the patients were advised against scratching the skin in the case of redness and swelling or small red blisters on the skin of the application site, and 75% alcohol was used for local disinfection.

All patients received nasal irrigation with normal saline thrice, and the duration of treatment was 1 month.

### 2.5. Observation Indicators

#### 2.5.1. Baseline Patient Profile

The baseline patient profile of the patients such as age, gender, course of disease, BMI, smoking, drinking, and education level was recorded.

#### 2.5.2. Clinical Efficacy

With reference to *Allergic Rhinitis Diagnosis and Efficacy Evaluation Criteria* [15], the clinical efficacy of patients after treatment was evaluated. Efficacy = (total scores before treatment − total scores after treatment)/total scores before treatment × 100%. Curative effect index ≥66% is considered markedly effective, 26% ≤ curative effect index ≤65% is effective, and curative effect index ≤25% is ineffective. The total treatment efficacy = (effective + markedly effective)/total × 100%.

#### 2.5.3. Serum IgE Level

5 ml of fasting venous blood was collected from the patient before and after treatment. After anticoagulation and centrifugation, the serum IgE level of the patient was determined using the enzyme-linked immunosorbent assay.

#### 2.5.4. Nasal Mucosal Eosinophils (EOS)

A cotton swab was used to swab the patient's turbinate forward and backward 2–3 times, and the exfoliated cells of the nasal mucosa were smeared on the glass slide. The collected exfoliated cells of nasal mucosa were prepared for observation by paraffin embedding, dewaxing, hematoxylin-eosin staining, dehydration, xylene transparent, and neutral gum sealing, and the morphology of eosinophils was observed under light microscope. The EOS counts of 10 or more consecutive visual fields were carried out under high power field (40 × 10 x), and the average was taken to score.

#### 2.5.5. Syndrome Scores

① Sneezing: no more than 3 consecutive sneezes are recorded as 0 points, 3–9 consecutive sneezes are recorded as 1 point, 10–14 consecutive sneezes are recorded as 2 points, and 15 consecutive sneezes or more are recorded as 3 points. ② Running nose: 0 points indicate that the number of times to wipe the nose is less than 2 times daily; 1 point indicates that the number of times to wipe the nose is 2–4 daily; 2 points indicate that the number of times to wipe the nose is 5–9 daily; and 3 points indicate that the number of times to wipe the nose is 10 or more daily. ③ *Nasal Congestion*. 0 points: there is no need to breathe through the mouth; 1 point: the patient occasionally breathes through the mouth; 2 points: the patient frequently breathes through the mouth; and 3 points: the patient cannot breathe through the nose completely. ④ Itchy nose: 0 points indicate no itching, 1 point indicates occasional itching, 2 points indicate tolerable persistent itching, and 3 points indicate unbearable nasal itching.

#### 2.5.6. Physical Signs Scores

1 point: there is mild swelling of the lower nose; the middle turbinate and nasal septum are still visible; 2 points: the nasal septum is close to the inferior turbinate, and there are small gaps between the inferior turbinate and nasal septum; 3 points: the inferior turbinate is close to the nasal septum and the base of the nose, and no middle turbinate or middle turbinate mucosal polypoid changes can be seen.

#### 2.5.7. Serum Inflammatory Substances

Enzyme-linked immunosorbent assay was used to determine the serum interleukin-4 (IL-4) and interferon-*γ* (IFN-*γ*) levels before and after treatment.

#### 2.5.8. Incidence of Adverse Reactions

The adverse reactions during the treatment of the two groups of patients were recorded.

### 2.6. Statistical Analysis

GraphPad Prism 7 (GraphPad Software, San Diego, USA) was used to plot the graphics, and SPSS23.0 software was used for data analyses. The counting data are expressed as [n(%)] and analyzed using the chi-square test, and measurement data are expressed as (mean ± SD) and analyzed using students' *t*-test. Differences were considered statistically significant at *p* < 0.05.

## 3. Results

### 3.1. Baseline Patient Profile

The general data of the two groups of patients were not statistically different (*P* > 0.05) (Table 1).

### 3.2. Clinical Efficacy

In the control group, 14 cases were markedly effective, 16 cases were effective, and 10 cases were ineffective. In the research group, 23 cases were markedly effective, 14 cases were effective, and 3 cases were ineffective. Rupatadine fumarate plus acupoint application was associated with a significantly higher efficacy versus rupatadine fumarate alone (*χ*^2^ = 4.501, *p* = 0.034). (Figure 1).

### 3.3. Serum IgE Levels

The IgE levels of the two groups of patients after treatment significantly decreased, and the research group had lower results (*p* < 0.05). (Figure 2).

### 3.4. EOS Content

After treatment, the EOS content of the two groups of patients decreased, and the EOS content of the research group was significantly lower than that of the control group (*p* < 0.05, Figure 3).

### 3.5. Syndrome Scores

The research group had significantly lower syndrome scores than the control group (*p* < 0.05). (Table 2).

### 3.6. Vital Sign Scores

The physical sign scores of the two groups of patients were reduced after treatment, and the research group showed significantly lower results (*p* < 0.05) (Table 3).

### 3.7. Serum Inflammatory Factor Levels

Rupatadine fumarate plus acupoint application resulted in significantly lower IL-4 levels and higher levels of INF-*γ* versus rupatadine fumarate alone (*p* < 0.05). (Figures 4 and 5).

### 3.8. Incidence of Adverse Reactions

The two groups showed a similar incidence of adverse events (*p* > 0.05).

## 4. Discussion

Allergic rhinitis is an IgE-mediated inflammatory disease of the nasal mucosa, which is caused by exposure to allergens [16]. Thus, anti-allergy is an essential part of the treatment of the disease. It is documented that rupatadine fumarate tablets are a potent anti-allergic drug. Clinical research found that rupatadine fumarate relieved the clinical symptoms and signs of allergic rhinitis and reduces the infiltration of eosinophils in the nasal mucosa. Moreover, its combination with acupoint application can further improve curative effect of allergic rhinitis and mitigate the symptoms, suggesting that rupatadine fumarate plus acupoint application shows a desirable effect in the treatment of allergic rhinitis. Accordingly, this study was conducted to explore the application effect of rupatadine fumarate plus acupoint application in allergic rhinitis complicated diabetes patients admitted to our hospital.

Western medicine recognizes that the onset of allergic rhinitis is related to the patient's physique and allergens [17]. After the allergen enters the nasal cavity for the second time, it binds to IgE on eosinophils and releases a large number of mediators such as leukotrienes and histamine to induce tissue edema and eosinophil infiltration. In this regard, the prerequisite for clinical treatment of allergic rhinitis lies in the identification of the allergen [18]. Relevant experimental studies have shown that the anti-tissue activity of rupatadine fumarate is significantly better than that of commonly used drugs such as loratadine and cetirizine [19]. The drug can effectively inhibit the activity of eosinophils, mast cells, and neutrophils and suppress the release of cytokines, emanating outstanding effects on the treatment of allergic rhinitis and urticaria. In the present study, patients in the control group were treated with rupatadine fumarate alone for one month and its was found that their signs and symptoms were alleviated, and EOS, IgE levels, and inflammatory cytokines were all ameliorated, suggesting the outstanding clinical value of rupatadine fumarate in the treatment of allergic rhinitis, and the results are consistent with the previous studies.

Chinese medicine believes that the contributory factors for allergic rhinitis include chill and wind, insufficient *q*i, and evil invasion, leading to deficiency of the spleen, kidneys, and lungs. Acupuncture, acupoint application, and Chinese medicine decoctions are key treatment methods to consolidate the function of viscera and the body's immunity, thereby mitigating clinical symptoms [20]. In the present study, patients in the research group were treated with rupatadine fumarate plus acupoint application using medicinal cakes with corydalis yanhusuo, white mustard seeds, asarum, and kansui root as ingredients for anti-allergic treatment. Corydalis yanhusuo can promote blood circulation and invigorate lung *q,* white mustard seeds warm the lungs and eliminate phlegm, asarum can dispel the heat, and kansui root can eliminate phlegm and induce diuresis to alleviate edema [21]. The combination of the above herbs for acupoint application can warm *yang*, promote *qi*, dispel wind and chill, and clarify the nose and orifices. The results of the present study indicated that the acupoint application plus rupatadine fumarate can further enhance the therapeutic effect of allergic rhinitis and reduce the level of IgE, IL-4, and EOS activity. In addition, INF-*γ* inhibits the synthesis of IgE from B cells, and the patient's INF-*γ* level after treatment was significantly increased, indicating that acupoint application could effectively regulate the immune balance of patients with allergic rhinitis, reduce inflammation responses, and relieve clinical symptoms. The EOS content of nasal secretions in the research group of the patients after treatment was reduced, which is in line with the research results by Eocak et al. The limitation of this study lies in the absence of the exploration of the drug mechanism. More prospective randomized controlled studies are required for in-depth exploration of the possible mechanism to provide more evidence-based references for disease treatment.

## 5. Conclusion

Rupatadine fumarate plus acupoint application may offer a viable treatment alternative for allergic rhinitis complicated with diabetes as it alleviates the clinical symptoms, improves treatment efficiency, and enhances the anti-allergic effect of the drug, with a high safety profile. However, this study is a retrospective study, with a small sample size and short follow-up. Thus, further studies are required to evaluate the long-term efficacy of rupatadine fumarate plus acupoint application for the treatment of allergic rhinitis complicated with diabetes.

## Figures and Tables

**Figure 1:** Comparison of the clinical efficacy of the two groups of patients (*n* = 40,%).

**Figure 2:** Comparison of the IgE levels of the two groups of patients. *Note*. The abscissa indicates before and after treatment, and the ordinate indicates the level, IU/ml; the IgE levels of the control group before and after treatment were (204.63 ± 32.15) and (97.86 ± 14.15), respectively; the IgE levels of the research group before and after treatment were (205.55 ± 33.21) and (90.37 ± 13.47), respectively; ^*∗*^indicates that the IgE levels of the two groups of patients after treatment were significantly different (*t* = 2.425, *p* = 0.018).

**Figure 3:** Comparison of the EOS content of the two groups of patients.

**Figure 4:** Comparison of the serum IL-4 levels of the two groups of patients. *Note*. The abscissa indicates before and after treatment, and the ordinate indicates the detection level, pg/ml; the IL-4 levels of the control group before and after treatment were (78.93 ± 16.47) and (17.05 ± 4.21), respectively; the IL-4 levels of the research group before and after treatment were (79.06 ± 16.69) and (12.11 ± 3.35), respectively; ^*∗*^indicates that the IL-4 levels of the two groups of patients after treatment were significantly different (*t* = 5.807, *p* < 0.001).

**Figure 5:** Comparison of serum INF-*γ* levels of two groups of patients. *Note*. The abscissa indicates before and after treatment, and the ordinate indicates the detection level, ng/L; the INF-*γ* levels of the control group before and after treatment were (45.15 ± 10.75) and (55.63 ± 10.49), respectively; the INF-*γ* levels of the research group before and after treatment were (47.13 ± 11.02) and (68.27 ± 16.02), respectively; ^*∗*^indicates that the INF-*γ* levels of the two groups of patients after treatment were significantly different (*t* = 4.175, *p* < 0.001).

**Table 1:** Comparison of general information of the two groups of patients (*n* = 40).

	Control	Research	t/*χ*^2^	*P* value
Age (year)	30.53 ± 6.17	31.09 ± 7.11	0.376	0.708
Course of disease (year)	4.23 ± 1.21	4.16 ± 1.17	0.263	0.793
Gender			0.201	0.654
Male	22 (55)	20 (50)		
Female	18 (45)	20 (50)		
BMI (kg/m^2^)	24.16 ± 2.34	24.08 ± 2.27	0.155	0.877
History of smoking			0.457	0.499
Yes	24 (60)	21 (52.5)		
No	16 (40)	19 (47.5)		
History of drinking			0.800	0.371
Yes	18 (45)	22 (55)		
No	22 (55)	18 (45)		
Educational background			0.200	0.655
Middle school	11 (27.5)	10 (25)		
Middle school to high school	8 (20)	11 (27.5)		
High school or above	21 (52.5)	19 (47.5)		

**Table 2:** Comparison of the syndrome scores of the two groups of patients.

	Control (*n* = 40)		Research (*n* = 40)	
	Before treatment	After treatment	Before treatment	After treatment
Sneeze	2.38 ± 0.61	1.60 ± 0.59	2.41 ± 0.58	1.29 ± 0.44
t_control-research_/P_control-research_		2.664/0.0094		
Running nose	2.40 ± 0.54	1.44 ± 0.54	2.39 ± 0.52	1.09 ± 0.33
t_control-research_/P_control-research_		3.498/0.0008		
Nasal obstruction	2.09 ± 0.61	1.56 ± 0.35	2.13 ± 0.58	1.26 ± 0.43
t_control-research_/P_control-research_		3.422/0.001		
Rhinocnesmus	1.88 ± 0.35	1.55 ± 0.34	1.89 ± 0.37	1.14 ± 0.56
t_control-research_/P_control-research_		3.907/0.0002		
Total score	8.73 ± 1.31	6.18 ± 1.42	8.70 ± 1.27	4.87 ± 1.34
t_control-research_/P_control-research_		4.244/0.0001		

**Table 3:** Comparison of the physical sign scores of the two groups of patients.

Group	n	Before treatment	After treatment
Control	40	2.47 ± 0.55	1.53 ± 0.52
Research	40	2.46 ± 0.53	0.91 ± 0.42
t-value			5.866
*P* value			<0.001

## Data Availability

The data used to support the findings of this study are available from the corresponding author upon request.
